The article "Moderate carbohydrate, moderate protein weight loss diet reduces cardiovascular disease risk compared to high carbohydrate, low protein diet in obese adults: A randomized clinical trial" was published in 2008. Journal: Nutr Metab (Lond).

# Moderate carbohydrate, moderate protein weight loss diet reduces cardiovascular disease risk compared to high carbohydrate, low protein diet in obese adults: A randomized clinical trial

**DOI:** 10.1186/1743-7075-5-30

**Published:** 2008-11-07

**Authors:** Denise A Walker Lasker, Ellen M Evans, Donald K Layman

**Affiliations:** 1 Division of Nutritional Sciences, University of Illinois at Urbana-Champaign, Urbana, IL, USA; 2 Department of Kinesiology and Community Health, University of Illinois at Urbana-Champaign, Urbana, IL, USA; 3 Department of Food Science and Human Nutrition, University of Illinois at Urbana-Champaign, Urbana, IL, USA

## Abstract

**Background:**

To evaluate the metabolic effects of two weight loss diets differing in macronutrient composition on features of dyslipidemia and post-prandial insulin (INS) response to a meal challenge in overweight/obese individuals.

**Methods:**

This study was a parallel-arm randomized 4 mo weight loss trial. Adults (n = 50, 47 ± 7 y) matched on BMI (33.6 ± 0.6 kg/m^2^, *P *= 0.79) consumed energy restricted diets (deficit ~500 kcal/d): PRO (1.6 g.kg^-1^.d^-1 ^protein and < 170 g/d carbohydrate) or CHO (0.8 g.kg^-1^.d^-1 ^protein and > 220 g/d carbohydrate) for 4 mos. Meal challenges of respective diets were utilized for determination of blood lipids and post-prandial INS and glucose response at the beginning and end of the study.

**Results:**

There was a trend for PRO to lose more weight (-9.1% vs. -7.3%, *P *= 0.07) with a significant reduction in percent fat mass compared to CHO (-8.7% vs. -5.7%; *P *= 0.03). PRO also favored reductions in triacylglycerol (-34% vs. -14%; *P *< 0.05) and increases in HDL-C (+5% vs. -3%; *P *= 0.05); however, CHO favored reduction in LDL-C (-7% vs. +2.5%; *P *< 0.05). INS responses to the meal challenge were improved in PRO compared to CHO (*P *< 0.05) at both 1 hr (-34.3% vs. -1.0%) and 2 hr (-9.2% vs. +46.2%), an effect that remained significant after controlling for weight or fat loss (both *P *< 0.05).

**Conclusion:**

A weight loss diet with moderate carbohydrate, moderate protein results in more favorable changes in body composition, dyslipidemia, and post-prandial INS response compared to a high carbohydrate, low protein diet suggesting an additional benefit beyond weight management to include augmented risk reduction for metabolic disease.

## Introduction

Obesity is a significant risk factor for cardiovascular disease (CVD) [1,2]. The risk, at least in part, is related to abnormal blood lipids consisting of elevated triacylglycerides (TAG), low high density lipoprotein cholesterol (HDL-C), and small, dense low density lipoprotein cholesterol (LDL-C) particles. This lipid profile is considered an atherogenic dyslipidemia and recognized as a primary feature of Metabolic Syndrome (MetS), an established risk factor for CVD and type 2 diabetes mellitus (T2DM) [3].

Dyslipidemia and MetS are both associated with high habitual simple dietary carbohydrate intakes, reduced insulin (INS) sensitivity, and elevated post-prandial INS [3-6]. Evidence is accumulating that post-prandial glycemia is an important risk factor for CVD [7,8]. Reaven et al [4] reported that although hypertriacylglyceridemia is an essential component of MetS, it is secondary to post-prandial INS response in risk for CVD. Even in individuals with normal blood glucose response, post-prandial INS varied more than 4-fold and the greatest post-prandial INS responses (i.e. compensatory hyperinsulinemia) had the highest TAG concentrations. More recently, Krauss et al [9] reported a linear relationship of carbohydrate intake and prevalence of atherogenic dyslipidemia in healthy subjects.

Reducing carbohydrate intake with replacement of either fat or protein has been shown to reduce TAG and increase HDL-C even under weight stable conditions [4,9,10]. Substitution with protein may be more beneficial than fat for lipid changes [9-13] and improvement in INS action [5,14,15]. Indeed, independent effects of protein on glycemic regulation [16,17] suggests protein may be a more effective dietary change than increases in fat intake for reducing risk for metabolic disease.

In this context, the aim of this study was to compare the relative efficacy of two weight loss diets differing in macronutrient content on fasted TAG and post-prandial INS in response to a meal challenge in overweight or obese individuals. We compared the conventionally accepted USDA Food Guide Pyramid diet (CHO) with a moderate carbohydrate, moderate protein (PRO) diet. Macronutrients for both dietary treatments fall within the Acceptable Macronutrient Distribution Range (AMDR) established by the Institute of Medicine's (IOM) Dietary Reference Intakes (DRI) [18]. We hypothesized that the PRO weight loss diet would result in greater fat mass loss and more favorable changes in post-prandial INS response and features of dyslipidemia compared to an isocaloric CHO diet.

## Methods

### Design

This study was a parallel-arm randomized 4 mo weight loss trial. Subjects were blocked on gender, matched on age (47.2 ± 1.0 y, *P *= 0.52), BMI (33.6 ± 0.6 kg/m^2^, *P *= 0.79) and fasting glucose (5.4 ± 0.1 mmol/L, *P *= 0.24). Diet treatments consisted of a PRO diet (carbohydrate ~40%; protein ~30%; fat ~30%) or an isocaloric CHO diet (carbohydrate ~55%; protein ~15%; fat ~30%).

### Subjects

Eighty-seven adults were interviewed for participation. Sixty-five adults aged 40 to 56 y were enrolled to participate in the weight loss study. Exclusion criteria were BMI < 26 kg/m^2^, body weight > 140 kg [due to dual energy X-ray absorptometry (DXA) scanning bed constraints], smoking, any existing medical conditions requiring medications that could impact primary or secondary outcomes of the study, and use of oral steroids or anti-depression medications. Reported results are based on n = 50 (M = 19; F = 31), due to either lack of adherence to protocol or loss to follow-up at 4 mo and one subject started training for a marathon (n = 15; PRO = 7; CHO = 8). The study was approved by the Institutional Review Board at the University of Illinois at Urbana-Champaign. All subjects gave written informed consent prior to participation.

All subjects participated in a baseline evaluation period that included a 24-h food recall, instructions for weighing and recording of foods, two 3-d weighed food records during separate weeks and measurements of weight, height, and blood lipids. This evaluation period from first contact with subjects was 10 to 20 d and served as an initial control period for each subject. During this baseline period, subjects were instructed to maintain stable body weight and consume a diet similar to the past 6 mo. After the baseline period, subjects reported to the nutrition research laboratory at 0630 h after a 12 h overnight fast for weight measurement and blood collection.

### Diet Treatments

Similar to our previous studies [11,14,19], the prescribed CHO diet provided dietary protein at 0.8 g.kg^-1^.d^-1 ^and > 220 g/d carbohydrate (~15% and ~55% of energy intake respectively). The prescribed PRO diet provided dietary protein at 1.6 g.kg^-1^.d^-1 ^and < 170 g/d carbohydrate (~30% and ~40% of energy intake respectively). Dietary lipids were constant between diets (~30% energy intake). These diets were designed to fall within the AMDR established by the IOM with minimum intakes for carbohydrates at 130 g/d and protein at 0.8 g.kg^-1^.d^-1 ^and upper limits for carbohydrates at 65% and protein at 35% of total energy intake [18]. The two diets were formulated to be equal in energy (7100 kJ/d; 1700 kcal/d), total fat intake (~57 g/d) and fiber (~14 g/1000 kcal^-1^.d^-1^). Each group received a menu plan with meals for each day meeting established nutritional requirements [18] and dietary lipid guidelines [20]. Diet differences between groups were designed to reflect direct substitution of foods in the protein groups (meats, dairy, eggs and nuts) for foods in the refined grain/starch groups (breads, rice, cereals, pasta and potatoes). Education guidelines for the CHO group followed USDA *MyPyramid *[21] and emphasized restricting dietary fat and cholesterol with use of whole grain breads, rice, cereals and pasta. For the PRO group, education guidelines emphasized use of high quality proteins including lean meats, dairy and eggs. Both diets included 5 servings/d of vegetables and 2 to 3 servings/d of fruit.

### Education Program and Monitoring

Subjects were provided electronic food scales and instructed to weigh foods at all meals. Subjects documented a 3-d weighed food record for each week throughout the study. Nutrient intakes were evaluated as mean daily intakes from 3-d weighed records using Nutritionist Pro software (First DataBank Inc. 2003, San Bruno, CA). After baseline data collection, subjects received instructions from a research dietitian about their specific diet including menus, food substitutions, portion sizes, and procedures for maintaining weighed diet records. Throughout the 4 mo study, subjects were required to attend a 1 h meeting each week at the nutrition research facility. Meetings were specific for each treatment group and directed by research dietitians who provided diet and exercise information and reviewed diet records for treatment compliance. Each week, subjects were weighed in light clothing without shoes and provided 3-d weighed food records.

The education program focused on diet compliance with minimal guidance regarding exercise. Activity guidelines emphasized lifestyle recommendations for physical activity based on NIH Guidelines for Weight Management [22]. These guidelines recommend a minimum of 30 min of walking 5 d/wk. Participation in physical activity for the groups was voluntary. Physical activity was monitored using daily activity logs and 3 d/mo subjects wore armband accelerometers (BodyMedia, Cincinnati, OH). Activity logs were collected each week. Records indicated that subjects exercised ~90 min/wk with no difference between diet treatment groups (*P *> 0.05).

### Body Weight and Composition

Body weight was measured using an electronic scale (Tanita, Model BWB-627A, Tokyo Japan). Whole body composition was determined by DXA (Hologic, QDR4500A, Bedford MA) and scans for a given individual were analyzed by the same technician using standard manufacturer guidelines. The CVs for DXA outcomes of interest in our laboratory are ~1.5%.

### Meal Challenge and Blood Measurements

Subjects came to the nutrition research facility after a 12 h fast at baseline and 4 mo for venous collection of fasted and 1 h and 2 h post-prandial blood. At baseline, all subjects consumed the CHO meal challenge (energy = 1656.77 kJ, protein = 15.32 g, carbohydrate = 55.35 g, lipid = 13.33 g, saturated fatty acid (SFA) = 7.63 g, cholesterol = 38 mg, and fiber = 2.93 g) that resembled their pre-study dietary composition. After 4 mo treatment and adaptation to the diets, subjects consumed the meal challenge of their respective diet treatments, i.e. CHO (composition listed above) or PRO (energy = 1662.94 kJ, protein = 33.24 g, carbohydrate = 28.18 g, lipid = 16.57 g, SFA = 7.26 g, cholesterol = 307.41 mg, and fiber = 1.05 g). Serum total cholesterol (TC), HDL-C and TAG were determined by standardized methods [23] by Washington University School of Medicine Core Laboratory for Clinical Studies (St. Louis, MO) with LDL-C calculated using the Friedewald equation [24]. Plasma insulin (MP Biomedicals, Irvine, CA; catalog # 07260105) was determined by a commercial RIA kit. Plasma glucose (ThermoTrace, Noble Park, Victoria AUS; catalogue # TR15498) was determined by glucose oxidase. The intra-assay CVs for insulin and glucose were 5.5% and 1.5% respectively.

### Statistics

The primary dependent variable in this study was change in 2 h post-prandial INS; therefore we determined our statistical power using this outcome. Previous work in our laboratory [14,25] determined INS responses to a meal challenge in the PRO group were reduced by 85% whereas the CHO group was reduced by 50% (and effect size between groups of ~1.0) in response to 10 weeks of weight loss. With this anticipated effect size, an alpha (significance) level of 0.05 and a power of 90%, a sample size of 22 subjects per group would be required to find statistical differences in 2 h post-prandial INS between the PRO and CHO groups should it exist. Given an estimated retention rate of 75% based on previous weight loss studies, it was planned to recruit a minimum of 60 individuals into the study. Differences among groups at baseline were evaluated using a *t*-test. Primary outcome variables were post-prandial INS and TAG. All other evaluated data were secondary outcomes of interest. Log transformations of INS and TAG concentrations were used to acquire normal distributions. The primary analysis, conducted to evaluate the relative impact of diet treatment on these variables, utilized repeated measures ANOVA (*time *× *diet*). Due to fasted INS differences, we also performed a sub-set analysis with subjects matched on fasted INS. To evaluate treatment effects on primary outcomes controlling for changes in body composition, an ANCOVA was used where indicated. Homeostasis Model Assessment of insulin resistance (HOMA1-IR) was calculated using the formula (G_0 _× I_0_)/22.5 [26]. Percentage change was calculated as (((post-test)-(pre-test)/(pre-test)) × 100). A *P *value of < 0.05 was considered significant. Values are presented as means ± SEM. All data analyses were performed using SPSS version 15.0 (SPSS, Inc., Chicago, IL).

## Results

### Subjects

Baseline characteristics were similar for subjects in both treatment groups (*P *> 0.05) with exception of fasted INS (*P *= 0.04) (Table 1).

**Table 1:** Baseline body composition and metabolic characteristics of adult subjects ^1^

**Group**	**PRO (n = 25)**	**CHO (n = 25)**
Height (cm)	168.9 ± 2.3	168.2 ± 1.8
Weight (kg)	96.6 ± 3.9	94.3 ± 2.1
BMI (kg/m^2^)	33.8 ± 1.1	33.4 ± 0.7
Fat mass (kg)	35.2 ± 1.8	36.3 ± 1.8
Percent fat mass (%)	36.4 ± 7.7	38.2 ± 6.9
Glucose (mmol/L)	5.3 ± 0.2	5.5 ± 0.1
Insulin (pmol/L)	169.7 ± 19.7*	119.2 ± 13.7*
HOMA-IR	5.70 ± 0.74	4.09 ± 0.45
Total Cholesterol (mmol/L)	5.33 ± 0.19	5.52 ± 0.17
LDL-C (mmol/L)	3.41 ± 0.16	3.49 ± 0.13
Apolipoprotein B (mmol/L)	2.89 ± 0.15	2.80 ± 0.11
LDL-C/Apolipoprotein B ratio	1.21 ± 0.05	1.26 ± 0.04
HDL-C (mmol/L)	1.14 ± 0.07	1.27 ± 0.07
Triacylglyceride (mmol/L)	1.72 ± 0.18	1.66 ± 0.17

^1 ^Values are means ± SEM. * Indicates group difference, *P *< 0.05.

### Dietary Compliance

Daily menus were designed to provide energy for F = 7.1 MJ/d (1700 kcal) and M = 7.9 MJ/d (1900 kcal); however, subjects were free-living and ultimately determined final daily energy intakes. Weekly 3-d weighed food records indicated reductions in energy intake were similar between groups. Summary of dietary intake throughout the 4 mo period illustrates how subjects applied the two diets during intervention (Table 2). Consistent with research design, PRO consumed greater protein (~1.40 g/kg vs. ~0.77 g/kg) and less carbohydrate compared to CHO. Total dietary fat remained similar between the two diets. A treatment effect was present with a greater reduction in SFA (*P *= 0.02) and cholesterol (*P *= 0.001) in CHO vs. PRO. Additionally, fiber was increased from baseline in both groups with a trend for a greater increase in the CHO group (PRO ~8.2% vs. CHO ~35.8%; *P *= 0.08).

**Table 2:** Dietary intakes for adults at baseline and during weight loss protocol (4 mo)^1^

	Dietary Intake		*P *value ^2^
**Group**	**PRO**	**CHO**	
Energy (kJ/d)			
Baseline	9952 ± 566	9147 ± 486	
4 mo	6607 ± 235	5875 ± 391	>0.10
Protein (g/d)			
Baseline	94.5 ± 6.2	87.9 ± 5.5	
4 mo	121.4 ± 4.8	66.7 ± 2.9	<0.001
Carbohydrate (g/d)			
Baseline	291.7 ± 17.4	264.9 ± 16.6	
4 mo	152.6 ± 7.3	215.4 ± 12.3	<0.001
Fat (g/d)			
Baseline	90.4 ± 6.4	81.5 ± 5.4	
4 mo	56.2 ± 2.2	39.2 ± 2.9	>0.10
Saturated Fat (g/d)			
Baseline	30.8 ± 2.4	27.6 ± 2.1	
4 mo	22.6 ± 0.8	11.9 ± 1.0	<0.05
Cholesterol (mg/d)			
Baseline	298.6 ± 36.5	242.8 ± 25.6	
4 mo	348.8 ± 25.2	122.1 ± 12.0	<0.001
Fiber (g/d)			
Baseline	19.5 ± 1.9	17.9 ± 1.6	
4 mo	21.1 ± 1.9	24.3 ± 2.0	<0.10

^1 ^Values are means ± SEM; n = 25, PRO; n = 25, CHO for the sum of 3-d weighed records obtained at wk 4, 8, 12, and 16.

^2 ^*P *values represent *time *× *diet *interaction after 4 mo. No significant baseline differences were present.

### Body Weight & Composition

Both groups decreased body weight, BMI, and fat mass during the 4 mo treatment period. There was a trend (*P *= 0.07) for PRO to lose more body weight (-9.1 ± 0.9 kg) than CHO (-6.9 ± 0.8 kg) with a corresponding reduction in BMI (3.1 ± 0.3 kg/m^2 ^vs. 2.4 ± 0.3 kg/m^2^; *P *= 0.07). Changes in body composition indicated weight loss was predominately fat mass and PRO reduced fat mass more than CHO (-6.0 ± 0.6 kg vs. -4.4 ± 0.5 kg, respectively; *P *= 0.06). In addition, a greater reduction in percent fat mass was observed in PRO vs. CHO (-8.7% vs. -5.7%; *P *= 0.03).

### Fasted Glucose and Insulin

No effect of dietary treatment was evident in fasted plasma glucose (PRO = -0.28 ± 0.13 mmol/L vs. CHO = -0.52 ± 0.12 mmol/L; *P *= 0.19). However, differential diet responses occurred for fasted plasma INS with a reduction in PRO compared to an increase in CHO (*P *= 0.03; Figure 1A). Furthermore, after controlling for change in weight or fat mass, the treatment effect on fasted INS favoring the PRO group remained a trend (*P *= 0.07). Similarly, dietary treatment effect on HOMA-IR produced a decrease from baseline in the PRO group and an increase in the CHO group producing a trend for a treatment effect (-1.1 ± 0.7 vs. +0.4 ± 0.4; *P *= 0.08).

**Figure 1:** **Change in insulin concentration**. Change in insulin concentration, pmol/L, from baseline to 4 mo at fasted (**A**) 1 hr (**B**) and 2 hr (**C**) post-prandial in response to the meal challenge for adults consuming either the PRO (n = 25, gray bar) or CHO (n = 25, white bar) diet. Values are means ± SEM. *Indicates *time *× *diet *interaction *P *< 0.05.

### Post-prandial response to the Meal Challenge

Dietary treatment did not alter plasma glucose at 1 h (*P *= 0.39) or 2 h (*P *= 0.59) post-prandial (data not shown); however, PRO produced lower INS responses at 1 h (-34.3% vs. -1.0%; *P *= 0.005; Figure 1B) and 2 h (-9.2% vs. +46.2%; *P *= 0.011; Figure 1C) compared to CHO. Furthermore, reduced post-prandial INS effects in PRO remained after controlling for change in weight (1 h *P *= 0.013, 2 h *P *= 0.04) or fat mass (1 h *P *= 0.015, 2 h *P *= 0.04). As expected, in the CHO group, change in weight or fat mass were related to change in INS at 1 h post-meal challenge [r = 0.48 (*P *= 0.03) and r = 0.40 (*P *= 0.05)], respectively; however, the relation was not present at 2 h post-meal challenge [r = 0.28 (*P *= 0.18) and r = 0.30 (*P *= 0.14)]. Relations of the changes in the PRO group were not as robust with the strongest relation being an r = 0.23 between change in weight and change in INS at 2 h post-meal challenge (*P *> 0.27).

### Baseline insulin group difference: ANCOVA and matched subset analysis

Due to differences in fasted plasma INS between treatment groups after randomization (*P *= 0.04), we utilized a subset analysis on treatment groups matched on fasted plasma INS at baseline (n = 22, PRO = 139.2 ± 14.3 pmol/L; n = 22, CHO = 129.3 ± 13.7 pmol/L; *P *= 0.47) and with an ANCOVA controlling for baseline INS. Within the INS matched subset, the diet effect on fasted INS after 4 mo was no longer evident (*P *= 0.31); however, favorable effects of the PRO diet remained post-prandially at 1 h (PRO = -299.5 ± 69.7 vs. CHO = -165.0 ± 74.2; *P *= 0.02) and 2 h (PRO = -126.0 ± 57.1 vs. CHO = 9.2 ± 32.4; *P *= 0.03). Likewise, the ANCOVA results supported favorable post-prandial effects of the PRO diet (1 h, *P *= 0.02; 2 h, *P *= 0.04, respectively).

### Serum Lipids

At randomization serum lipid concentrations were similar among groups (Table 1). After 4 mo, serum lipid profiles changed in both groups; however, the patterns of change were affected by diet. There was a trend for greater decreases in TC in the CHO group compared to the PRO group (-0.39 ± 0.09 mmol/L vs. -0.13 ± 0.13 mmol/L; *P *= 0.09). LDL-C, Figure 2A, was reduced in the CHO group compared to an increase in the PRO group (-6.5% vs. +4.9%; *P *= 0.046). Both treatment groups exhibited a small (~11%) decrease in apolipoprotein B (ApoB) concentration at 16 wks that was not significantly different from baseline for the PRO or CHO group (*P *= 0.61; -0.41 ± 0.12 mmol/L vs. -0.33 ± 0.10 mmol/L). However, the decrease in ApoB coupled with the decrease in LDL-C in the CHO group produced a greater increase in the LDL-C/ApoB ratio, Figure 2B, in the PRO group compared to the CHO group (+22.0% vs. +7.3%; *P *= 0.045). HDL-C concentrations, Figure 2C, changed in opposite directions with an increase in PRO (+6.9%) and a decrease in CHO (-1.7%; *P *= 0.045). Reductions in TAG, Figure 2D, were greater in the PRO group (-26.8%), than in the CHO group (-7.0%; *P *= 0.01), an effect that remained after controlling for changes in both weight (*P *= 0.04) and fat mass (*P *= 0.04). When further exploring change in weight or fat mass in relation to this primary lipid outcome, there was a relation between TAG and weight and fat mass in the PRO group [r = 0.41 (*P *= 0.04) and r = 0.34 (*P *= 0.097)] respectively; however no relation was present in the CHO group [r = 0.019 and r = 0.029 (both *P *> 0.93)].

**Figure 2:** **Fasted serum lipid concentrations**. Change in fasted serum lipid concentrations, mmol/L, of LDL-C (**A**), LDL-C/ApoB ratio (**B**), HDL-C (**C**), and triacylglyceride (**D**), from baseline to 4 mo for adults consuming either the PRO (n = 25) or CHO (n = 25) diet. Values are each individual's data point (X) with means (black line bar) within each group. All outcomes had a *time *× *diet *interaction *P *< 0.05 between group means.

## Discussion

The PRO diet produced greater reductions in fat mass and a trend for greater weight loss compared to the CHO diet. Furthermore, the PRO diet produced greater improvement in features of dyslipidemia and post-prandial INS response. In support of our hypothesis, this study demonstrates that free-living overweight or obese individuals have greater reductions in risk factors for CVD and T2DM by utilizing a PRO weight loss diet instead of a conventional CHO diet. Specifically, the PRO diet modulates post-prandial INS and fasted TAG, two key risk factors and early markers for MetS, T2DM, and CVD.

The importance of these two markers, post-prandial INS and fasted TAG, is beginning to be appreciated in the clinical setting. Loss of post-prandial glucose control has been implicated as the first step of deterioration in individuals with MetS and T2DM. Deterioration of glycemic regulation often first appears as compensatory hyperinsulinemia seen post-prandial to a meal to maintain glucose uptake into cells and normal homeostasis [27]. In addition, dietary carbohydrate, specifically simple sugars, promote atherogenic dyslipidemia, mostly resulting from effects on TAG metabolism [9,28], thereby increasing risk of CVD.

In the current study, post-prandial INS response was determined after a mixed meal challenge similar in concept to that of an oral glucose tolerance test. The post-prandial response demonstrated a significant decrease in 1 h and 2 h INS in the PRO treatment (see Figure 1) which remained significant irrespective of weight or fat mass reduction. This positive outcome in response to the PRO diet is similar to results reported for other reduced carbohydrate diets [5,15]; however, the present study evaluated free-living overweight/obese individuals without diabetes and dietary fat was similar in the two dietary protocols. Regarding the most similar population, subjects with mild, untreated T2DM, the net mean 24 h integrated insulin and glucose area response was significantly decreased after 5 wk on a low carbohydrate diet compared to a high carbohydrate diet [15]. Moreover, our previous study utilizing a highly controlled diet design in which meals were provided to subjects resulted in similar adaptations in the post-prandial INS response [14]. This accumulating literature indicates that PRO diets are effective in improving post-prandial INS responses in free-living populations, supporting use of this diet treatment in reducing risk for MetS, T2DM, and CVD.

Likewise, fasted INS demonstrated a favorable response in PRO compared to CHO as seen by the significant decrease in fasted INS from baseline (see Figure 1) in addition to a decreasing trend in HOMA-IR. These two parameters along with the post-prandial INS responses suggest an increase in INS sensitivity in individuals consuming the PRO diet. These findings support the hypothesis that the macronutrient composition of weight loss diets, specifically exchanging protein for carbohydrate, minimize need for peripheral glucose uptake and improve insulin sensitivity (16).

High TAG, low HDL-C and high small dense LDL-C are components of atherogenic dyslipidemia commonly seen with MetS which also contributes to risk for CVD [29]. Consistent with reduced post-prandial INS, the PRO diet produced greater improvement in dyslipidemia. Serum TAG reduction was favored in PRO over CHO (see Figure 2) which was in agreement with previous studies in our lab [11,19] in addition to other clinical studies investigating weight loss protocols with reduction in dietary carbohydrate [5,9,12,13,15,30,31]. HDL-C increases in PRO (see Figure 2) are also in agreement with previous research using reduced carbohydrate diets [11,30-32]. Reductions in LDL-C in the CHO diet likely reflect consumption of half the amount of cholesterol and saturated fat compared to PRO due to increased consumption of animal protein sources in PRO although both lipid and saturated fat amounts decreased from baseline in both groups (see Table 2). Additionally, previous research has shown that LDL-C particle size increases with low carbohydrate diets, which is indicative of larger non-atherogenic LDL-C particles [9,31,33,34]. Using the LDL-C/ApoB ratio as an indication of particle size [35], this study found a significant increase in PRO compared to CHO (see Figure 2) suggesting a benefit of PRO on LDL-C particle size.

This study confirms that reducing dietary carbohydrates produces improvements in characteristics of dyslipidemia and insulin sensitivity [36]. Reducing carbohydrate intake can be achieved through energy restriction or replacement of carbohydrates with protein [9,11] or fat [10,31,33,34]. The relative merit of substitution with protein or fat remains unknown. McAuley et al [10] reported that changes in TAG, HDL-C and fasting insulin were similar with high protein or high fat diets but found greater improvements in LDL-C with the high protein diet. Likewise, PRO diets may have greater effects on satiety [17] and body composition [17,37]; however well-designed studies are required to elucidate this question.

This study is not without limitations. First, it must be taken into consideration that although we matched groups on fasted glucose, we did not match on fasted INS resulting in a statistical difference at baseline in this variable. To address this situation, we performed a subset analysis matching groups on fasted INS and used an ANCOVA controlling for baseline INS at 1 h and 2 h. These secondary analyses attenuated differences in fasted INS response to dietary treatment at 4 mo; however differences in post-prandial INS after the meal challenge remained. Second, exercise was not a mandatory part of the weight loss regimen and subjects averaged less than 100 min/wk of added exercise. Finally, subjects were free-living individuals and ultimate food choices were made at their discretion.

## Conclusion

In summary, this study evaluated diet specific outcomes of free-living overweight or obese subjects without diabetes. Subjects on either isocaloric diet complied with the prescribed protocol and reduced both weight and fat mass; however, the PRO diet was better overall than the CHO diet for risk reduction of metabolic disease beyond that of weight management. Greater improvements in post-prandial INS were demonstrated in subjects consuming the PRO diet with effects observed at 1 h and 2 h after a meal challenge. Additionally, fasted INS further supported the decrease in HOMA-IR for improvement in INS sensitivity in the PRO group. Features of atherogenic dyslipidemia improved significantly in the PRO group as demonstrated by decreases in TAG and increases in HDL-C and LDL-C/ApoB ratio. Collectively, these results support use of PRO diets with moderate carbohydrate, moderate protein over conventional CHO diets with high carbohydrate, low protein for decreasing risk for obesity, and more importantly, MetS, T2DM, and CVD. Future research is needed to 1) define optimal diet composition for individuals varying in risk for metabolic disease (e.g. hypercholesterolemia vs. MetS and 2) determine cellular mechanisms by which differing macronutrient diets produce these favorable health outcomes.

## Competing interests

DKL received grant/research support from the funding agencies for this research: the National Cattleman's Beef Association, The Beef Board and Kraft Foods.

## Authors' contributions

Design and development of this clinical trial conducted at the University of Illinois at Urbana-Champaign nutrition research laboratory was performed by DKL and EME. EME and DAL were responsible for the statistical analysis. DAL prepared the manuscript.
